# Design for Bedridden Elderly: Presenting Pressure Ulcer Product Design Based on Anthropometric Characteristics

This article has been retracted.

**DOI:** 10.1155/2022/4895038

**Published:** 2022-07-30

**Authors:** Jie Zhou, Wanqiang Li, Hong Hu

**Affiliations:** ^1^College of Art and Design, Beijing University of Technology, Beijing 100124, China; ^2^Haier Open Partnership Ecosystem, Qingdao Haier Intelligent Technology R&D Co., Qingdao 266000, China; ^3^School of Art and Design, Guangdong University of Technology, Guangzhou 510000, China

## Abstract

Pressure ulcers are a type of injury that causes tissue ischemia, a deficiency of nutrition and oxygen to the tissues, and, eventually, tissue necrosis when an area of skin is placed under constant pressure for an extended length of time. With the acceleration of the aging process, the problem of providing care for pressure ulcers for the bedridden elderly becomes increasingly urgent. This study conducts a field survey based on the research status of 221 disabled elderly in 16 communities on 7 typical streets in Beijing, focusing on the problem of pressure ulcer complications caused by bedridden. An automatic inflatable airbag mattress is designed according to anthropometric dimensions of bedridden elderly, pressure ulcer-prone areas, and the decompression standard, so that the airbag mattress can reduce the pressure in its initial shape. To achieve accurate control of the pressure in the pressure-prone areas of an airbag, air pressure control system is proposed which can control airbags individually and link multiple airbags, evaluating the safety of pressure ulcer points based on the data from sensors and making corresponding air pressure changes to reduce the possibility of generating pressure ulcers. The proposed pressure ulcer preventing system will be an efficient healthcare tool for families who had elderly bedridden patients, patients with chronic degenerative disease side effects, and terminal and postsurgical patients, as well as femur fractures, in their homes.

## 1. Introduction

Pressure ulcers, a serious and common complication, place a tremendous burden on the quality of life of older adults. Pressure ulcers are localized injuries to the skin or subcutaneous tissue at the bone eminence under pressure or combined shear or friction [1]. The treatment and nursing of pressure ulcers have been a challenge in the nursing field. The incidence of pressure ulcers in the bedridden elderly is high and shows a linear upward trend which is about 17.4% in elder people. In China, more than 20% of the elderly require care and attention in their daily lives, where 20% to 50% of the patients requiring long-term care suffer from pressure ulcers. Pressure ulcers have a long healing period and are painful and the elderly are prone to infection and even systemic failure as they gradually worsen [2].

The causes of pressure ulcers are complex including internal and external factors. Internal factors mainly include general health, mobility, nutritional status, skin moisture, age, prior history of pressure ulcers, medication history, and perfusion/oxidation-related problems. The external factors are divided into pressure, shear, skin microenvironment (heat and humidity), and friction [3]. Among the external factors, pressure is the most important factor causing pressure sores, especially in the rough projections of the human skeleton, where short periods of high-load damage are as damaging as long periods of low-load damage [4]. Various forces such as pressure, shear, and friction acting together are the most common causes of pressure ulcers and pose the highest risk to vulnerable patients, which can cause stress and strain when this happens. Friction and shear forces do not cause pressure ulcers alone, but can contribute to and aggravate pressure ulcers [5]. Pressure ulcers are likely to occur in elderly bedridden patients with other indications of contact surfaces in pressure and lack of adipose tissue protection, no muscle wrapping or thin muscle layer at the bone augmentation, with the key points being pressure, bone augmentation, and the absence of decompression tissue. The external pressure is mainly concentrated at the bony prominence, and the pressure on the human body in the supine or sitting position ranges from 1.33 to 6.66 kPa [6].

According to the Sixth Population Census and the 2010 China Aging Development Statistical Bulletin, by the end of 2010, China had fully entered the elderly society, with about 33 million bedridden and fully bedridden elderly in urban and rural areas. By the year 2022, there will be more than 42 million bedridden elderly and more than 29 million elderly who are over 80 years old, accounting for a total of 30% of the total elderly population. With the deepening of the degree of aging, the number of bedridden elderly will undoubtedly increase year by year; along with the extension of the life expectancy of the elderly [7], the prevalence and incidence of chronic and recuperative diseases have increased significantly and rapidly [8], and various reasons have led to the bedridden elderly with chronic diseases becoming a common phenomenon. It is increasingly difficult to meet the nursing service needs of the bedridden elderly, which must be complemented by equipment and facilities that are more adaptable to home and community-based elderly care [9].

Currently, products and services targeting the elderly involve dozens of industries, including nursing, rehabilitation, and finance, offering products and services such as clothing, food, housing, transportation, entertainment, and healthcare [10, 11]. Research on elderly products focuses on product development and design activities, that is, elderly product design methods and technical evaluation; research on age-appropriate technologies is reflected in different technical fields, such as Gates, Fisher, and Cooke, who study fall detection, prevention technology, and its products. Haux et al. [12] studied the use of ICT to help the elderly live and meet their healthcare needs. Heerink et al. [13] pointed out market-oriented suggestions from the perspective of the innovation process and innovation environment optimization. According to Hu et al. [14], wearable smart devices for the elderly pay more attention to multiproduct health tracking tools for the elderly. Classified by their static or dynamic nature, many advanced low-tech and high-tech support surfaces and overlays are available for patients bound to lie in bed for long periods. Static surfaces (such as foam-filled mattresses, air-filled mattresses, and fluid-filled mattresses) do not require electrical power, while dynamic surfaces (such as alternating air pressure mattresses or pneumatic ripple beds) require electrical power for shifting and redistributing the pressure within the surface [15, 16]. Iaizzo [17]stated that other integrated electronic beds like air fluidized beds and electronic moving air mattresses require high technology and heavy machinery to let air and ceramic sphere particles support the object on a stream mechanically. Frederick Shelton et al. [18] concluded that the best pressure distribution effects are from air cushions by comparing standard hospital-used spring foam cushions, high-quality foam, and low air pressure loss air cushions in a test. Although inflatable cushions and mattresses are widely used to reduce the external pressure on the body area, they are usually controlled by straight tube strips with automatic control, and air pumps control inflation and discharge to regularly switch the hardness of tubular strips to achieve the function of pressure management [19].

Therefore, this study chooses to prevent pressure ulcers caused by bedridden as the design goal and develop a mattress that can effectively reduce the incidence of pressure ulcers in the bedridden elderly. A new type of self-inflating airbag mattress is designed composed of multiple elastic airbags made of porous materials. To achieve accurate control of the pressure in pressure-prone areas, an airbag air pressure control system is proposed for reducing the local pressure caused by body weight, which evaluates the safety of pressure ulcers points based on the data returned by pressure and humidity sensors and makes corresponding air pressure changes for pressure sore-prone points in different areas to reduce the possibility of generating pressure sores.

The rest of the manuscript is organized as: Section 2 provides a detailed description of the proposed method. In Section 3, the process of airbag designing is illustrated and the different steps required for airbag design are presented.  Section 4 is about the discussion and the conclusion is presented in Section 5.

## 2. Methods

### 2.1. Research Process

The most common air mattresses on the market now do not subdivide the applicable population and ignore the particularity of the elderly under the advantage of versatility [20]. To minimize the pressure on the bone protruding part of the bedridden elderly in the supine state, the airbag mattress needs to have the ability to reduce the pressure of the pressure ulcer sites in its initial form; that is, the shape of the airbag corresponding to each part of the human body accords with the ergonomics of the elderly, increases the contact area between the airbag mattress and the human body, and reduces the pressure per unit area of the human contact surface. Therefore, this paper studies the anthropometric data of the elderly and the weight and pressure of various parts of the human body [21]. As shown in Figure 1, the proposed research process is as follows.

In the preparation phase, the following steps are performed:

- Analysis of the core needs of the main users and stakeholders, i.e., the bedridden elderly, their caregivers, and their families, and determining the prevention of pressure ulcers as the main design goal.
- Conducting theoretical research and definition of key issues, including characteristics of bedridden elderly, characteristics of pressure ulcers, elements of formation, major pressure sore producing sites, and existing research on pressure ulcer prevention products.
- Based on the combination of design objectives and the existing research, the functional requirements of the product are determined to regulate the pressure factors, microenvironment, and duration of pressure in the bedridden elderly, to increase the contact surface between the human body and the bed surface through soft and elastic materials, and to reduce the pressure per unit area, so that the weight of the human body is not excessively concentrated on the protruding part of the bone to achieve the purpose of pressure ulcer prevention.

In the design phase, the following steps are performed.

- Determining the specific data for each design element, including pressure factors, decompression criteria, and ergonomic data for the elderly.
- Identifying the materials, airbag size, etc. of the product in conjunction with research on hyperplastic materials and human scale.
- Controlling the airbag on the mattress individually, as it is necessary to match the airbag air pressure control system, design the airbag control system, the composition, and connection of the pneumatic device, and determine the inflation and deflation process.

### 2.2. Decompression Data Collection

According to the analysis of pressure ulcer formation factors and the Bergstrom conceptual model, the form factors of pressure ulcers are pressure and tissue tolerance, with the pressure factor depending on the intensity and duration of pressure and the tissue tolerance being influenced by internal factors (the patient's condition) and external factors (the microenvironment). Regarding external factors, the American Pressure Sore Advisory Committee [20] concluded that external factors (microenvironment) refer to the temperature of the skin surface or tissues, the relative humidity of the air, and the fluids on the skin surface (sweat, incontinence, wound drainage, moisture from the skin stratum corneum, etc.), with the airflow having a greater effect on skin surface temperature and humidity. Internal factors cannot be directly affected by design, so external factors are the design direction of this paper, namely, pressure factors (compression intensity and duration) and microenvironment (skin surface temperature, skin surface fluid, and air relative humidity).

#### 2.2.1. Pressure Standard

In 1930, Eugene Landis proposed that “the maximum pressure that normal human skin capillaries can withstand is 32 mmHg,” which is currently accepted as the golden rule in medical care and scientific research [5] and the relationship between external pressure and duration in etiology and pathology of ischemic ulcers shows that external pressure of 600 [mmHg] within 1 hour or 150 [mmHg] within 12 hours can cause stress ulcers. The normal skin capillary pressure is 2.7 kPa, and plethysmography is used to measure the normal capillary pressure from 2.1 kPa to 4.3 kPa. If the pressure exceeds 4.3 kPa, the pressure will block capillary perfusion to the tissue, resulting in skin blood flow arrest, and metabolic waste will contribute to tissue degeneration followed by tissue ischemia and necrosis [21, 22]. Pressures below 4.67 kPa for more than 4 h, or while keeping the pressure constantly changing, do not change the tissue even when the pressure reaches 25.3 kPa for up to 1 h. However, irreversible damage may result when the skin tissue is continuously exposed to pressures above 9.33 kPa for more than 2 h [23]. Therefore, the airbag mattress focuses on sensitive adjustment of the skin pressure value and needs to make the patient contact with the mattress after the pressure peak of the bony prominence is less than 32 mmHg for the standard.

#### 2.2.2. Microenvironment Standard

The increase in local skin temperature increases the oxygen consumption of the body's basic metabolism and aggravates the hypoxia of the pressurized part, which will increase the incidence of pressure sores to a certain extent. Sae-Sia et al. [24] found by monitoring patients with a nerve injury that the skin temperature of the sacrococcygeal region increases by 1.2°C before the development of pressure ulcers, so monitoring of elevated body temperature was used as a trigger indicator to determine whether the temperature microenvironment of bedridden elderly exceeded safe values. Kokate et al. [16] defined subhypothermia as mild to moderate hypothermia between 28 and 35°C. Due to the decreased sensitivity of thermoreceptors in the elderly, the ability of body temperature regulation and heat dissipation will also decrease. Therefore, the contact temperature of the bedridden elderly can be maintained at mild hypothermia.

When the skin is infiltrated excessively, the tissue becomes soft and fragile [25]. The incidence of pressure ulcers in patients with incontinence is about 5 times that in patients without incontinence. Due to the high accuracy of the measurement of water content in the stratum corneum of the skin and limited measurement methods, this study adopted the method of increasing the contact area between the skin and the air to adjust the humidity of the local microenvironment of the skin.

### 2.3. Calculation of Anthropometric Data of the Elderly

In terms of the dimensions of the airbag mattress for preventing pressure ulcers, the most important thing is the size of the airbags based on the ergonomics set corresponding to each pressure ulcer occurrence point. First, divide the human body according to the pressure ulcer occurrence point; then, as a product for bedridden elderly, the anthropometric dimensions of the elderly are calculated. Next, combined with the division of the human body and the anthropometric dimensions of the elderly, the specific dimensions of each region are calculated, respectively. In terms of the pressure dimension of the pressure ulcer prevention airbag mattress, it is necessary to obtain the weight of the body tissue in each area, simulate the relationship between the human body and the airbag pressure, and divide the area of the human body according to the standard mannequin and the pressure ulcer points to obtain the approximate contact area and body tissue weight, as shown in Figure 2.

#### 2.3.1. Anthropometric Data and Application of the Elderly

To design and study the products for the bedridden elderly, the first step is to define the anthropometric data of the elderly, so that the basic product form meets the ergonomics of the elderly and generates low-pressure values in the head, shoulder blade, back, sacrum, thigh, and heel [26]. The back, sacrum, thighs, and heels of the five parts of the bone protrusions all produce small pressure values. According to China's national standard GBl000-88, considering the main dimensions of the human body in standing and sitting postures, the division of each area is shown in Figure 3.

*(1) Univariate/1D approaches using 5th–95th percentile values*. The body dimensions of any particular group of objects conform to the law of normal distribution; that is, most of them belong to intermediate values, and only a small number belong to values that are too large and too small, which are distributed at both ends of the range. P5, P50, and P95 are common percentiles, with “P5” representing the “small” size, which means that 5% of the population is less than this value. The “P50” represents the “medium” size, which means that 50% of the population is more or less than this size, and “P95” represents the “large” size, which means that 95% of the body dimensions are less than this value [26]. According to the design requirements and the national standard of adult body dimensions in China, the body dimensions of standing and sitting posture of P5, P50, P95, and P99 are for men aged 36 to 60 years and females aged 36 to 55 years. The physiological status of the elderly changes significantly with age [27], such as loss of height and weight [28]. At present, research on body dimensions of the elderly has not been widely conducted in China; and since body dimensions of the elderly tend to stabilize after reaching the age of 65 [29], there is no need for further subdivision of body dimensions of the elderly. Since people become smaller with age and the height of most elderly people is 5% shorter than when they were young, the height dimensions of the elderly in this design were reduced by 5% from the national measured dimensions (GB 10000–88, 1988). The estimated main dimensions of the elderly for P5, P50, P95, and P99 can be derived as shown in Table 1.

According to Figures 4–10, to divide the longitudinal human body area, the algorithm for dividing each part of the longitudinal dimension is as follows. GB/T 5703 defines the basic items, terms, and definitions of anthropometry. And the calculation in Algorithm 1 are cited from GB/T 5703.

According to Figure 4 for the longitudinal and transverse divisions of body areas, the values of longitudinal and horizontal dimensions of each body area were calculated as shown in Table 2, with partial reference to the Japanese AIST body size database (AIST,1991–92) due to the small number of horizontal dimension measurement dimensions of the national standard anthropometric measurements. To make this design applicable to most people, two groups of P50 (including P1, P5, and P10) and below P99 (including P95 and P99) are used for the values of body size, and the initial values required for the calculation are the red parts.

#### 2.3.2. Calculation and Application of Elderly Body Pressure

In this study, the principle of decompression airbag is used, so the calculation of human body pressure mainly focuses on the relationship between the human body and the airbag. When the human body is in contact with a solid surface, it presents the most basic stress-strain relationship. When the fluid in a confined space acts on a wall of *A*_*s*_ [*m*^2^] area or a virtual plane with a uniformly distributed compression force *F*[*N*], as shown in Figure 5(a), the pressure P[*N*/*m*^2^] is calculated as follows:

(1) $$\begin{array}{c} p=\frac{F}{A_{s}}. \end{array}$$

Since the gas is a compressed fluid and its density hardly changes with temperature, when a solid of weight *w*[Kgf] is placed on the airbag, as shown in Figure 5(b), the pressure generated by the solid acts equally on all parts of the airbag, which is expressed as the following equation according to Pascal's theorem:

(2) $$\begin{array}{c} P_{c}=\frac{w}{A_{0}}=\frac{F_{0}}{A_{s}}=p_{0}, \end{array}$$

where *p*_*c*_ denotes the contact pressure,  *A*_*c*_ denotes the contact area, and *F*_0_*p*_0_ denotes the total pressure and the internal pressure of the airbag, respectively. It can be derived from (2) that the contact pressure *p*_*c*_ can be directly measured by measuring the internal pressure *p*_0_, and it can be controlled by changing *p*_0_.

In the human supine state, this design uses airbags to minimize the skin pressure caused by body weight. When the human body weight is constant, the body pressure can be minimized only by increasing the contact area between the human body and the airbag surface; so when the weight and contact area of the body parts are known, the optimal pressure that minimizes the pressure on human skin is *P*_*i*_, as given in (3), where *w*_*i*_*A*_*i*_ represents the mass and contact area of each body part.

(3) $$\begin{array}{c} P_{i}=\frac{w_{i}}{A_{i}}. \end{array}$$

Based on the study of a standard human mannequin by D.A. Winter [30] and the study of general human body measurement data by Inhyuk Moon [28] and others using an approximate mannequin, in this design, the human body is divided into five parts: head, shoulder and back, waist and hip, legs, and feet, i.e., *i* = head, shoulder and back, waist and hip, legs, and feet. *w*_*i*_*A*_*i*_ can be calculated from anthropometric data and approximate mannequin data, so the body pressure *P*_*i*_ of the *i* part of the body can be minimized by increasing *w*_*i*_. The length of each part is the relative length of the body height (h), and the approximate mannequin dimensions are shown in Figure 6.

According to the 4–13 approximate mannequin, the head and heel can be approximated as a sphere and the leg as a cylinder; then it is assumed that the maximum contact surfaces of the head, heel, and leg are hemispherical and semicylindrical, respectively, while the shoulder-back and waist-hip parts are approximated as rectangular and the contact area shape is rectangular. The approximate contact area is calculated as

(4) $$\begin{array}{c} A_{\text{Head}}=2\pi \cdot 0.065{\text{h}}^{2},\\ A_{\text{Shoulder and back}}=0.240\text{h}\cdot 0.174\text{h,}\\ A_{\text{Waist and hip}}=0.253h\cdot 0.191h,\\ A_{leg}=2\pi \left(0.0275h\right)\left(0.329h\right),\\ A_{\text{feet}}=2\pi {\left(0.024h\right)}^{2}. \end{array}$$

Knowing the maximum contact area and the weight of body parts, the pressure on each contact surface can be calculated using (3). According to the anthropometric data of the elderly mentioned above, the approximate contact area with three heights of 170 cm, 180 cm, and 190 cm can be obtained, as shown in Table 3.

The approximate weights of different parts are shown in Table 4.

According to Tables 4 and 5 and to cover a broader range of people, if we take that the weights of the elderly are 65 kg, 75 kg, and 85 kg, respectively, then the corresponding approximate weights of 170 cm, 180 cm, and 190 cm are shown in Table 5.

## 3. Airbag Design

### 3.1. Design Guidelines

Based on anthropometric data and pressure calculations of various parts of the elderly, and taking into account the pathology of pressure ulcer formation, this study developed a design concept of medical auxiliary products for the prevention of pressure ulcers, reduced the pressure on the joint surface by lowering the force and decreasing the area and duration of the joint surface, optimized the back skin contact environment by using structural materials such as heat dissipation and ventilation, accurately measured the pressure at the joint points with the help of sensors, and provided feedback to reduce the pressure at vulnerable areas.

In the product form and structure design path of the airbag mattress for pressure ulcers prevention, to avoid pressure ulcers to the greatest extent, the airbag mattress needs to fit the human body to the greatest extent. Therefore, the core technical points of this product are as follows:

- The longitudinal height, transverse dimension, shape, and distribution of the airbag.
- Airbag pressure value to avoid pressure ulcers.
- The material of the airbag suitable for the body of the elderly and the pressure demand of the airbag.

The longitudinal height of the airbag is calculated by ergonomics, the horizontal size of the airbag can be determined by anthropometry, and the shape and distribution of the airbag can be determined by medical studies on the shape of human bones and muscles [29]. According to the approximate human mannequin, the weight of different parts and the contact area with the airbag can be determined; thus, the pressure value of the airbag in different parts can be determined, and the filling capacity of the airbag can be determined. Therefore, the appropriate airbag material can be selected according to the pressure demand.

In the product technology path of airbag mattresses for pressure ulcers prevention, the formation of pressure ulcers is affected by pressure, microenvironment, and duration, which can be measured by pressure sensors, temperature and humidity sensors, and timers, respectively. Pressure ulcers are formed on the head, shoulder blades, buttocks, and heels, so it is possible to determine where the sensor is buried. The functional requirements of the product in this study are that it can ensure that no pressure ulcer occurs when the pressure intensity of less than 4.7 kPa does not exceed 4 h and the pressure intensity of less than 9.3 kPa does not exceed 2 h. To keep the weight of the human body from being concentrated on the bony prominence, the area of the contact surface between the human body and the bed is increased, so that the pressure per unit area is reduced, and the pressure can be controlled within a safe range to prevent pressure ulcers.

### 3.2. Design of Pressure Ulcer-Proof Airbag Mattress

The conceptual design of the scheme is carried out according to the functional requirements, with a total of 6 schemes, as shown in Figure 7. The final design is determined after iteration of option 1 and option 5, modeled, rendered, product details as shown in Figure 8.

Figure 9 shows the connection, relationship, and arrangement of the pneumatic device of the automatic inflatable airbag mattress. The airbag is nested on the airbag fixing ring, which is convenient to fix the position of the airbag on the one hand and can avoid excessive deformation of the airbag in the process of inflating and discharging [30]. The airbag bottom bracket supports the airbag and the lower part of the airbag fixing ring, which makes the airbag and the mattress more integrated, avoids displacement inside the mattress, and also facilitates the connection of the airway, the trachea, and the airbag. The airway is located below the airbag bottom bracket to store excess gas during inflation and deflation, and the soft air tube connects the airway and the airbag in series. The mattress integrates the airbag, the airbag fixing ring, the airbag bottom support, and the airway; the hardware equipment of the airbag air pressure control system is set inside the mattress; and the rest of the space is filled with materials such as latex, and the user can directly use the automatic inflatable airbag mattress. The automatic inflatable airbag mattress is controlled by the airbag pressure control system and is composed of five parts of airbags corresponding to different parts of the human body. The airbag pneumatic device consists of an airbag air pressure control system (PLC, pressure sensor), airway, motor, and air pump. The airbag air pressure control system is connected to the automatic inflatable airbag mattress through an air tube connected to the airway and the farthest end of the airbag in the shared airway is provided with a pressure sensor to detect the air pressure and feedback to the airbag pressure control system. The airbag pressure control system controls the solenoid valve installed on the trachea to adjust the airbag inflation and discharge to reduce joint pressure and prevent pressure ulcers. The use of an internal quick-connect safety connector to connect the airbag mattress and the air pump can effectively prevent throat loosening or air leakage.

For the length and width of the mattress, considering the height of the elderly and the length of the bed, the length of the airbag mattress for preventing pressure ulcers is divided into three sizes: 170 cm, 180 cm, and 190 cm. The product research in this study is designed with the height of the elderly at 170 cm and below. After the dimensional calculation, the data of each area of the human body division and the overall dimensions of each part are appropriately rounded and proportionally adjusted to obtain the main dimensions and processing dimensions of each part of the antipressure sore module mattress.

As for the thickness of mattresses, according to market research, common mattresses are spring mattresses, palm mattresses, latex mattresses, water mattresses, angular sloping spine mattresses, air mattresses, and magnetic mattresses. A larger proportion of spring mattresses can be roughly divided into continuous spring, independent spring, and partition spring. The partitioned spring mattress designed for the head, neck, shoulder, rib, waist, vertebral tail, buttocks, legs, and feet of the human body is the most ergonomic type of spring mattress and is consistent with the purpose of ergonomics in this paper. Therefore, in addition to taking into account the space for internal control hardware, the thickness of the preventing pressure ulcer airbag mattress mainly refers to the thickness of the partition spring mattresses circulating on the market. Mattress thickness is usually 200 mm, 220 mm, 240 mm, and 260 mm, which also includes the thickness of the bedding layer such as latex, sponge, memory material, or brown. The airbag mattress in this design can be divided into two parts: the airbag and the mattress body, and the thickness of the mattress body is the height of the airbag, the bed surface, the bottom support plate, and the control hardware composed of the air pump, motor, controller, and airway as shown in Figure 10. The height of the irregularly shaped airbag following the curve of the human body varies, and to achieve the effect of preventing pressure ulcers, part of airbags are higher than the bed, so the height of the airbag in the main part of the mattress is taken to be the smallest, i.e., 82 mm, airbag part, to avoid the pressure caused by the weight of the elderly lying flat on the airbag mattress to compress the control hardware at the bottom of the mattress; the use of a 10 mm bottom support plate and side support frame made of brown can help the airbag to maintain its shape and reduce the pressure on the bottom hardware, which can reduce the thickness of the mattress body. The volume and height of the control hardware depend mainly on the air intake and exhaust volume of the airbag, and a small miniature air pump can be used. Therefore, it is estimated that 200 mm of the main part of the mattress can meet the demand, as shown in Figure 10.

As shown in Figure 11, this design is based on ergonomics, according to the previous functional division of the human body, through different forms of airbags corresponding to the human body structure, with particular attention to the head, scapula, hip (hip), and foot (hind heel) decompression at the joints. According to the medical statistics on the site of pressure ulcers, the airbags are corresponding to the pressure ulcer points. Airbag A0 corresponds to the head, airbag B corresponds to the scapula, airbag C corresponds to the waist, airbag *D* corresponds to the hip, A1, A2, A3, A4 corresponds to the spine, A4 corresponds to the sacrum, airbag E corresponds to thigh, airbag F corresponds to knee fossa, airbag G corresponds to the calf, and airbag H corresponds to heel. Based on the height and weight statistics of the elderly, anthropometric data, and approximate anthropometric mannequins, the size and shape of the airbag are designed to correspond to the human body structure to fit the human body to the maximum extent possible.

### 3.3. System Design Based on PLC

This study is based on the pressure sensor to design a control system that can adjust the pressure adaptively. This control system can switch the air inlet and outlet of the airbag bed pump and then automatically pressurize and depressurize to achieve the function of timely pressure adjustment, the core of which is the Programmable Logic Controller (PLC). PLC is an electronic system of digital operations specially designed for applications in industrial environments, which adopts programmable memory and can store and execute operation instructions such as logic operation, sequence control, timing, counting, and arithmetic operation to control various types of mechanical devices or production processes through digital or analog inputs and output [31].

To calculate the pressure on the airbag, it is necessary to determine the volume of different types of airbags first. The airbag volume can be calculated according to the dimensions of each airbag in Figure 10, as shown in Table 4.

According to the approximate contact area of the elderly in Tables 4 and 5, the approximate contact area of each airbag can be calculated. Based on the volume, the weight capacity, contact area of each airbag, and the medically prescribed pressure threshold of the skin capillaries, the pressure threshold for monitoring each airbag pressure sensor in the airbag mattress can be derived, and the feedback from the controller is prescribed accordingly. The airbag mattress pneumatic device prevents pressure ulcers by reducing local pressure peaks. The air pressure control system of the airbag mattress is shown in Figure 12 which can adaptively reduce the local body pressure of the bedridden elderly of different heights and weights to prevent pressure ulcers. The airbag mattress device consists of nineteen airbags made of porous material, which allows air leakage to help reduce temperature and humidity, and reducing peak pressure, temperature, and humidity helps to reduce the development of pressure sores. To determine the optimal airbag pressure for each user, this design divides the body parts into five parts: head, shoulder blades, waist and hip, legs, and feet. Then, based on the anthropometric data of height and weight and an approximate mannequin, the pressure of each part is calculated independently from the weight of each part. The control system uses PLC as the main controller, the PLC collects the pressure signal of pressure sensors, the temperature and humidity signal of temperature and humidity sensor, and the time signal of the timer and then sends a signal to the relay to control the action of the electromagnetic reversing valve after calculation and comparison to achieve the purpose of controlling the airbag inflation, deflation, and pressure maintenance.

The principle of the airbag mattress device is shown in Figure 13. First, a set of pressure detection modules is designed. Its function is to use the pressure sensor to measure the pressure between the body and the airbag when different body areas are on the different softness of the airbag. Then the pressure is converted into the change of the voltage value by the partial voltage circuit; after reading the change of the voltage value, the value is transmitted to the IPC industrial computer through RS-232; last, write pressure change parameter threshold in PLC. The air pump stores the gas in the airway, when it is necessary to adjust the pressure of different airbags on the airbag mattress, the PLC issues instructions after judging according to the pressure change parameter threshold and opens the solenoid valve of the corresponding airbag; then the prescribed airbag will use the airway to inflate and deflate, to achieve the function of timely automatic adjustment of pressure and reduce the skin pressure of the human body to prevent pressure ulcers.

The pneumatic device of the airbag mattress is shown in Figure 14. Sn(*n* = 0,1,2,3,4,5,6,7) denotes the air pressure sensor, V23-n (*n* = 0,1,2,3, 4,5,6,7) shows the two-position three-way reversing valve, V22-n (*n* = 0,1,2,3,4,5,6,7) is the two-position two-way reversing valve, Mn (*n* = 0,1,1 2,3,4,5,6,7) represents the silencer, Sn (*n* = 0,1,2,3,4,5,6) denotes the commutator, and AP is the air pump. The current position of the reversing valve in the figure is the initial position when the high-pressure air flows into the airbag and the airbag is inflated. When the two-position three-way reversing valve operates and the two-position two-way reversing valve does not operate, the gas in the airbag is discharged through the two reversing valves, and the pressure in the airbag decreases. When the two-position three-way reversing valve and the two-position two-way reversing valve operate at the same time, it is the pressure-holding state; at this time, the high-pressure air from the air pump will not flow into the airbag, and the gas in the airbag will not be discharged into the air.

Under the stressful condition, the flow of airbag inflation and deflation for the four areas of the head, shoulder blades, waist and hip, legs, and feet, which are prone to pressure ulcers when the patient is lying down, is shown in Figure 15. When A0 (the head) pressure sensor detects that the pressure exceeds the normal threshold, the A0 airbag will deflate moderately to reduce the pressure, while the A1 and A2 airbags will inflate moderately to increase the bearing force of the neck and spine parts. When the pressure sensors on the left and right sides of B (the shoulder blades) airbags detect that the pressure exceeds the normal threshold, the two B airbags will deflate moderately to reduce the pressure, while the A1/A2/C airbags will inflate moderately to increase the upper spine and lumbar bearing force. When the pressure sensors on the left and right sides of D (the hip) airbags detect that the pressure exceeds the normal threshold, the two D airbags will deflate moderately to reduce the pressure, while the A3/A4/C airbags will inflate moderately to increase the lower spine and lumbar bearing force. When the pressure sensors on the left and right sides of the H (the feet) airbags detect that the pressure exceeds the normal threshold, the 2 H airbags will deflate moderately to reduce the pressure, while E \ F \ H airbags will inflate moderately to increase the leg bearing force.

The system implementation flow of the airbag pneumatic device is determined according to Figure 15 inflation and deflation process. First of all, during the initial process of the system, each airbag will be inflated to a set initial pressure value. Then examine in turn whether the airbag pressure values of different parts of the human body are within the range of the safety threshold.

- S1: to judge whether the airbag A0 (the head) air pressure is too high, if it exceeds the safety pressure threshold, open the two-dimensional three-way valve and two-position two-way valve of airbags A1 and A2, and let the gas in the airway enter into the airbag to pressurize the airbag. Airbag A0 only opens the two-position three-way valve, letting the gas in the airbag enter the airway when the airbag decompression. If the airbag A0 (the head) air pressure does not exceed the safety pressure threshold, then proceed to the next stage.
- S2: if the airbag A0 (the head) air pressure is normal, then judge whether the airbag B air pressure corresponding to the scapula is too high. If it exceeds the safety pressure threshold, open the two-dimensional three-way valve and two-position two-way valve of airbags A1, A2, and C, let the gas in the airway enter into the airbag to make the airbag pressurized, make the airbag of cervical vertebra, thoracic vertebra, and waist bulge moderately to bear more pressure; and airbag B only opens the two-position three-way valve, and let the gas in the airbag enter into the airway with the airbag decompression. If the airbag B (the shoulder blades) air pressure does not exceed the safety pressure threshold, then proceed to the next stage.
- S3: if the air pressure of airbag B (the shoulder blades) is normal, then check whether the airbag D (the hip) pressure is too high. If it exceeds the safety pressure threshold, open the two-dimensional three-way valve and two-position two-way valve of the airbags A3, A4, and C, so that the airbags of the lumbar spine and waist are properly bulged to bear more pressure; airbag D only opens the two-position three-way valve to decompress the airbag when the gas in the airbag enters the airway. If the airbag D (the hip) pressure does not exceed the safety pressure threshold, then proceed to the next stage.
- S4: if the airbag D (the hip) pressure is normal, then judge whether the airbag H (the heel) pressure is too high. If it exceeds the safety pressure threshold, open the two-dimensional three-way valve and two-position two-way valve of airbags E, F, and G, so that the airbags of the thigh, leg fossa, and calf bulge moderately to bear more pressure. Airbag H only opens the two-position three-way valve, so that the airbag decompresses when the gas in the airbag enters the airway. If the airbag H pressure does not exceed the safety pressure threshold, then keep the same.
- Repeat the 4 stages of S1–S4.

The components are connected to form a principle model, such as the pneumatic device model controlled by PLC is as shown in Figure 16.

## 4. Discussion

This study conducted a survey on the vulnerability and care services needs of the urban disabled elderly in Beijing for more than one year. The basic characteristics of 221 users were that 80% were 70–90 years old, 60% were female, more than 60% did not have a partner, more than 60% depended on their partners or children to care for them, and nearly 50% were living in small 20–60-square-foot homes. In terms of health conditions, according to the tests of ADL and IADL scales, it was found that the current self-care ability (ADL mean score 3.8) of the surveyed elderly was low, and it was difficult to afford instrumental activities of daily living (IADL mean score 2.92), and the moderate to severe disability (ADL <4) was all concentrated in the elderly who are over 80 years old, and the completely disabled and incapacitated elderly were concentrated between 80 and 90 years of age. The willingness of the disabled to go to care institutions was highly related to the status of their cofamilies, and whether the elderly go to care institutions to a considerable extent represents the stability of their lives or sense of security. Elderly living with their mates will go to care institutions because their mates are also of an old age and lack care ability, but more than 60% of the elderly people were unwilling to go to institutions for the aged when they have a choice. There was no doubt that the family structure of elderly people living alone and senior couples will make the plight of elderly home care more and more prominent. In the process of the construction of community home care service, the singleness and lack of home care products will undoubtedly increase the difficulty of nursing and the pain of the elderly, and the entry point of choosing to prevent pressure ulcer mattresses is precise because of its high application value for the bedridden elderly [32].

Society's understanding of aging is gradually deepening, from “Healthy Aging” to “Positive Aging” to “Productive Aging,” which both indicate that the needs of the elderly are no longer single, and complex scenarios, diverse needs and optimized experiences all put higher requirements on aging design. Emerging technologies are increasingly used in all kinds of aging designs, which needs to combine ethnography, participatory design, and real-life evaluation, to explore the design and use of technologies for promoting the social life of seniors [33]. Abundant research on aging designs with the use of technologies exists on the many assistive technologies that provide help with everyday physical and cognitive tasks. In recent years, with the use of artificial intelligence, AR/VR/MR, 5G, robots, new energy, and other emerging technologies, the design related to “Positive Aging” makes the life of the elderly develop intelligently and efficiently; e.g., digital strategies, such as telemedicine and e-health, offer the potential to deliver positive aging in a cost-effective manner [34]. During the design process, a variety of diverse technologies in smart products for the seniors based on novel types of input, such as sensors and cameras, and interaction paradigms, such as voice, gaze, brain signals, and gestures, means that users (senior) and designers will be presented with more sophisticated alternatives among the several factors that influence technologies adoption. With the maturity of digital technology and hardware, sensors, ICT, distributed technology, and other technologies can be used to improve the quality of life and mental happiness of the elderly, and this paper uses sensors and PLC for operation control [35].

The first limitation of this paper is that this design is only for the pressure adjustment of the bedridden elderly in the supine state. The pressure ulcer-prone points in the supine, left and right lateral, sitting, and other states vary greatly, and the airbag shape is difficult to meet all postures. Secondly, the research on the human dimensions of the elderly has not been widely carried out in China, and the anthropometric data on the elderly lack more reliable and accurate data sources. This paper uses estimated data based on statistics and needs more reliable anthropometric data on the elderly in China as support. Finally, this paper designed products and control systems based on medical knowledge and anthropometric theory, and the validity of the design has not been verified by real-life test experiments or design simulations. In the future, contact sensors will be considered for human testing, or design simulations will be used to verify the efficiency of body pressure dispersion and also to test the medical feasibility by measuring the flow and pressure of blood.

## 5. Conclusion

Combined with the aging design strategy, aiming at the phenomenon of pressure ulcer complications occurring in the bedridden elderly, an intelligent airbag mattress is presented to prevent pressure ulcers by reducing the peak local pressure, and a matching airbag control system is designed. The airbag control system can synthesize the pressure values, pressure duration, and skin temperature and humidity values of pressure ulcer-prone points for analysis and inspection and prevent or eliminate pressure ulcers by controlling the inflation and deflation of airbags at relevant areas. The designed mattress minimizes the pressure on the skin caused by weight through the airbag, which is designed according to ergonomics and allows the waist and legs to share the stress, reducing pressure sores at the source. This design provides real-time pressure detection at pressure ulcer-prone points and accurately controls pressure values and duration at key points to extend the turning interval and reduce the possibility of pressure ulcers, greatly reducing the inconvenience of bedridden elderly' lives. However, the pressure ulcer prevention intelligent airbag mattress must also be tested and adjusted in real-world settings, including the adaptability of the airbag module distribution, size, and material for the elderly body, as well as the effectiveness of decompression and pressure ulcer prevention, the accuracy and fault tolerance of the coordinated feedback between the sensors, controllers, and the airbag, and the overall product safety evaluation.

## Figures and Tables

**Figure 1:** Design research process.

**Figure 2:** Calculation of Anthropometric Data of elderly.

**Figure 3:** Division map of each area of the human body.

**Figure 4:** Vertical and horizontal division of body parts.

**Figure 5:** Pressure variation of external load on airbag pressure. (a) Airbag internal pressure and (b) external contact pressure.

**Figure 6:** Approximate mannequin.

**Figure 7:** Conceptual design.

**Figure 8:** Scheme details.

**Figure 9:** Connection relationship of automatic inflatable airbag mattress.

**Figure 10:** Correspondence analysis between the airbag and human body.

**Figure 11:** Product applications.

**Figure 12:** Air pressure control system.

**Figure 13:** Airbag mattress pneumatic device.

**Figure 14:** Airbag mattress pneumatic device.

**Figure 15:** Airbag inflation and deflation process.

**Figure 16:** Model of a pneumatic device controlled by PLC.

**Algorithm 1:** Division of the longitudinal dimension.

**Table 1:** The body dimensions of China adults and elders at different percentages (mm).

Percentage		Adult body dimension								Elderly body dimension							
		Male 36–60				Female 36–55				Male 60–85				Female 55–85			
		P5	P50	P95	P99	P5	P50	P95	P99	P5	P50	P95	P99	P5	P50	P95	P99
	Weight/kg	49	61	78	85	44	55	70	76	49	61	78	85	44	55	70	76
	Height	1576	1667	1761	1798	1477	1560	1646	1683	1568	1659	1752	1789	1470	1552	1638	1675

Torso	Shoulder height	1278	1360	1445	1482	1191	1265	1343	1376	1272	1353	1438	1475	1185	1259	1336	1369
	Shoulder width	343	373	401	415	323	350	378	390	343	373	401	415	323	350	378	390
	Maximum head width	145	154	164	168	145	155	164	169	144	153	163	166	144	154	163	168
	Maximum shoulder width	398	433	473	489	368	405	449	468	398	433	473	489	368	405	449	468
	Width of chest	254	285	321	336	238	269	309	327	254	285	321	336	238	269	309	327
	Perineal high	724	784	846	875	668	726	784	810	721	780	842	871	665	718	780	806
	Sitting hip width	299	327	361	375	317	353	390	411	299	327	361	375	317	353	390	411

Limbs	Upper arm length	289	313	337	348	260	282	306	317	289	313	337	348	260	282	306	317
	Hand functional height	676	736	795	818	646	700	753	775	676	736	795	818	646	700	753	775
	Elbow height	950	1019	1087	1119	895	956	1018	1042	950	1019	1087	1119	895	956	1018	1042
	Thigh length	425	462	501	518	399	434	472	489	423	460	498	515	397	432	470	486
	Calf length	336	367	400	416	311	341	373	388	334	365	399	414	309	339	372	387
	Tibia height	407	441	478	493	375	407	441	456	405	439	475	490	374	405	439	454

**Table 2:** The division of each area of the human body and the horizontal and vertical dimensions of each part (mm).

		Male 60–85				Female 55–85			
Percentage		P5	P50	P95	P99	P5	P50	P95	P99

Weight/kg		49	61	78	85	44	55	70	76

Vertical dimensions	Height	1568	1659	1752	1789	1470	1552	1638	1675
	Head height	296	306	314	314	285	293	302	306
	Shoulder and back height	322	334	351	356	290	303	308	327
	Waist and hip height	274	283	292	301	250	256	265	267
	Hip height	229	239	245	248	230	238	238	236
	Waist height	45	44	47	53	19	18	27	31
	Thigh length	423	460	498	515	397	432	470	486
	Calf length	334	365	399	414	309	339	372	387
	Foot height	71	74	76	76	65	66	67	68

Horizontal dimensions	Maximum head width	144	153	163	166	144	154	163	168
	Shoulder width	343	373	401	415	323	350	378	390
	Lower scapula width	161	187	214	222	132	162	186	188
	Chest width	254	285	321	336	238	269	309	327
	Waist width	248	274	298	305	217	253	289	293
	Seated hip width	299	327	361	375	317	353	390	411
	Knee width	97	107	113	114	92	101	113	117
	Heel width	59	64	69	69	58	62	68	69

**Table 3:** The approximate contact area of the elderly (mm).

	170	180	190
Head	638	74035	851
Shoulder-back	1003	1165	1338
Waist-hip	1397	1566	1744
Legs	1643	1842	2052
Feet	87	101	116

**Table 4:** Approximate weight calculation of the elderly.

	Head	Shoulder-back	Waist-hip	Legs	Feet
Weight	0.081w	0.355w	0.342w	0.194w	0.028w

**Table 5:** Approximate weight of the elderly (kg).

	170	180	190
Head	5	6	7
Shoulder-back	23	27	30
Waist-hip	22	26	29
Legs	13	15	17
Feet	2	2	2

## Data Availability

Previously reported data of human dimensions of Chinese adults were used to support this study and are available at GB-10000-88, human dimensions of Chinese adults (S) 1988. These prior studies (and datasets) are cited at relevant places within the text as references (GB-10000-88, human dimensions of Chinese adults (S) 1988).
